# *In Vitro* Immunomodulatory Effects of *Inonotus obliquus* Extracts on Resting M0 Macrophages and LPS-Induced M1 Macrophages

**DOI:** 10.1155/2022/8251344

**Published:** 2022-04-21

**Authors:** Dayue Shen, Yating Feng, Xilan Zhang, Jing Liu, Le Gong, Hui Liao, Rongshan Li

**Affiliations:** ^1^School of Pharmacy, Shanxi Medical University, Taiyuan 030001, China; ^2^Department of Pharmacy, Fifth Hospital of Shanxi Medical University (Shanxi Provincial People's Hospital), Taiyuan 030012, China; ^3^Department of Nephrology, Fifth Hospital of Shanxi Medical University (Shanxi Provincial People's Hospital), Taiyuan 030012, China

## Abstract

**Background:**

*Inonotus obliquus* (Chaga) is a parasitic fungus that is distributed mainly in northeast China. Our literature research showed chaga polysaccharides have bilateral effects on tumor necrosis factor (TNF)-*α* and interleukin (IL)-1*β* levels when they exert antitumor and antidiabetic activities. The current research tried to explore the influence of chaga extracts on inflammatory factors via macrophage polarization which has bilateral immune-regulation not only on healthy tissue homeostasis but also on pathologies.

**Methods:**

Chaga was extracted with 100°C water and precipitated with 80% ethanol. The extracts were studied on RAW264.7 macrophage at resting condition (M0) and lipopolysaccharide (LPS)-activated subtype (classic activated macrophage, M1). The IL-1*β*, TNF-*α*, nitric oxide (NO) level, and the protein expressions of M1 and alternative activated macrophage (M2) markers including IL-1*β*, inducible NO synthase (iNOS), mannose receptor (CD206), and arginase (Arg)-1 were compared.

**Results:**

The 100 g extracts contained 13.7 g polysaccharides and 1.9 g polyphenols. Compared with M0, the 50 *μ*g/mL extracts increased NO level (*P* < 0.05) and decreased CD206 and Arg-1 expression significantly (*P* < 0.05). The extracts at 100–200 *μ*g/mL increased NO and TNF-*α* level (*P* < 0.05), but increased iNOS and IL-1*β* expression significantly (*P* < 0.05). Compared with M1, the extracts decreased NO level at 25, 50, 100, and 200 *μ*g/mL and decreased IL-1*β* and TNF-*α* level at 100–200 *μ*g/mL significantly (*P* < 0.05). At 25–200 *μ*g/mL, the extracts significantly increased CD206 and Arg-1 expression and decreased IL-1*β* and iNOS expression separately (*P* < 0.05).

**Conclusions:**

Our research suggested that the bilateral effects of the chaga extracts on iNOS, IL-1*β,* and NO level on M0/M1 macrophages might be related with chaga polysaccharides and chaga polyphenols. Some *in vivo* anticancer and antidiabetic research of purified chaga polysaccharides related to macrophage differentiation should be conducted further.

## 1. Introduction

*Inonotus obliquus*, also known as chaga, is a parasitic fungus that grows on birch trees and belongs to the Hymenochaetaceae family [1]. They are mainly distributed in northeast China and northern Russia [2]. Since the 16^th^ century, this fungus has been used as food and medicine for the prevention and treatment of malignant tumors, diabetes, and cardiovascular diseases in Russia, Poland, and the Baltic countries [3]. Chaga has biologically active substances such as polysaccharides, polyphenols, and flavonoids, and has various biological activities such as antitumor, hypoglycemic, antioxidation, and immune stimulation [4, 5]. Based on PubMed, Scopus, Wanfang database (Wanfang), and China National Knowledge Infrastructure (CNKI), an extensive literature survey was conducted about the research of chaga and its active substances on different diseases.  Figure 1(a) shows that most of the articles of chaga were on antidiabetes research, followed by anticancer research over the last 10 years (2012–2021). As the two main active ingredients in chaga, Figures 1(b) and 1(c) show that polysaccharides have more research papers than polyphenols in antidiabetes and anticancer research.

Both cancer and diabetes are immunology-related diseases [6, 7]. Cancer immunology is the most rapidly expanding field in cancer research with the emerging importance of immunity in cancer pathogenesis [6]. A potential immune-regulatory factor in cancer immunology might represent an alternative target for the treatment of cancers [8]. In the development of type 2 diabetes mellitus (T2DM), chronic inflammation plays an important role, and the proinflammatory environment maintained by the innate immunity, including macrophages and related cytokines, can be influenced by adaptive immunity [7]. Our further literature research detailed the relationships between immune-regulatory signaling pathways of chaga polysaccharides and their antidiabetic [9–14] and antitumor activities [15–21] in Figure 2.

From Figure 2, it was interesting to see the bilateral effects of chaga polysaccharides on the following cytokines: protein kinase B (Akt) and matrix metalloprotein-9 (MMP-9) levels were increased in antidiabetic activities [10, 12], but decreased in anticancer effects [18, 19]. Conversely, chaga polysaccharides decreased reactive oxygen species (ROS), interleukin (IL)-1*β*, and tumor necrosis factor (TNF)-*α* level in antidiabetic activities [9] but increased ROS, IL-1*β*, and TNF-*α* level in anticancer effects [16, 17]. Our previous study showed that both IL-1*β* and TNF-*α* are the markers of a classic activated macrophage (M1), which is polarized from resting macrophage (M0) by lipopolysaccharide (LPS) [22, 23]. Based on the above literature research and our previous study, we were interested in investigating the effects of chaga on different macrophage conditions such as M0 and M1 and thus inflammatory factors such as IL-1*β* and TNF-*α*.

Macrophages are bone marrow-derived leukocytes that are key for healthy tissue homeostasis but can also contribute to pathologies such as metabolic syndrome [24]. Broadly, a macrophage is divided into three phenotypes: M0, M1-like, and alternative activated macrophage (M2)-like [23]. M1 and M2 have different transcription profiles and act by eliminating bacteria, viruses, and fungi from the host or repairing the damage triggered by inflammation, respectively [25]. In this research, the protein expressions of two markers of M1 differentiation including IL-1*β* and inducible nitric oxide synthase (iNOS), and two markers of M2 polarization, mannose receptor (CD206), and arginase (Arg)-1 were determined by Western blotting, and the levels of IL-1*β*, TNF-*α*, and nitric oxide (NO) were also tested.

## 2. Materials and Methods

### 2.1. Preparation of Samples

Chaga was collected from Lvliang Mountains in Shanxi province. The process for chaga extracts is shown in Figure 3 and described briefly as follows.

The chaga was cut into coarse particles with a grain size of about 2-3 mm. The 1 kg chaga particles were soaked into 10 L distilled water (w/w: 1 : 10) at room temperature for 3 h and then boiled at hot water (100°C) [26] for 1 h. The supernatants were removed and the residue was extracted another two times for 30 min, respectively. The total supernatants were collected and precipitated by 80% ethanol (v/v) [27] at 4°C for 12 h. The precipitates were collected and dried at 0.07 MPa vacuum and 55 ± 1°C to a constant weight. These dried samples were used for further research on the contents of polysaccharides and polyphenols.

### 2.2. Analyses of Polysaccharides Content

#### 2.2.1. Standard Curve of Total Sugar

The total sugar was tested with phenol-sulfuric acid method using glucose as the standard [28]. About 1.0 mg/mL D-glucose (Solarbio, Beijing) stock solution was pipetted in deionized water at final concentrations of 25, 30, 35, 40, 45, 50, 55, and 60 *μ*g/mL in 2 mL total volume and mixed with 2 mL of 5% phenol solution (v/v) and 10 mL of concentrated sulfuric acid (Shidande, Shanghai, P.R. China) separately. The mixture was placed in a water bath at 80°C and kept for 30 min. It was then cooled to room temperature, and the A values were measured at 486 nm using a spectrophotometer (Persee, Beijing). The standard curve of total sugar was obtained using the A value as the ordinate and the concentration as the abscissa.

#### 2.2.2. Standard Curve of Reducing Sugar

The reducing sugar was determined by 3,5-dinitrosalicylic acid (DNS) assay [29]. 50 mg of glucose (Solarbio, Beijing) was weighed accurately and dissolved in 100 mL deionized water, and 0.5 mg/mL glucose standard solution was prepared. Then 0.0, 0.6, 0.8, 1.0, 1.2, and 1.4 mL of the prepared glucose standard solution were added to 2.0, 1.4, 1.2, 1.0, 0.8, 0.6 mL deionized water, respectively, and mixed with 1.5 mL DNS (Shidande, Shanghai, P.R. China) reagent separately. The mixtures were boiled in a water bath at 100°C for 5 min, then quickly cooled with running water, and diluted to 10 mL, and the absorbances were measured at a wavelength of 540 nm. A standard curve of reducing sugar was drawn using glucose concentration as the ordinate and absorbance as the abscissa.

#### 2.2.3. Determination of Polysaccharide Content

The dried extract was accurately weighed and dissolved in deionized water, and 0.2 mg/mL solution of the extract was made separately. Then, 2 mL of the 0.2 mg/mL solution was mixed as aforementioned. The values of the total sugar and the reducing sugar were calculated according to the standard curve obtained above. Finally, the total polysaccharides content was calculated from the reducing sugar subtracted from the total sugar.

### 2.3. Analyses of Polyphenol Content

Polyphenol content was analyzed using Folin–Ciocalteu method, which was optimized by response surface methodology [30]. Briefly, 20 *μ*L of 1 mg/mL extract was mixed with 100 *μ*L of Folin–Ciocalteu's reagent and 1,580 *μ*L of 50% EtOH. The above mixture was kept for 10 min in the dark. Then, 300 *μ*L of an aqueous solution of 0.2 g/mL Na_2_CO_3_ was added and put back in the dark for 2 h with continuous stirring. Finally, the mixture was centrifuged at 10,000 g for 3 min and 200 *μ*L of the extract was put in a Greiner microplate (Solarbio, Beijing). The absorbance was measured with the Infinite M200 PRO microplate spectrophotometer (Tecan Trading AG, Switzerland) at 765 nm. The polyphenol content was calculated according to a calibration curve made using gallic acid as the analytical standard.

### 2.4. Cell Source and Culture

The mouse macrophage RAW264.7 cell line was purchased from the Procell Life Science & Technology Co., Ltd. (Wuhan, China). According to the instructions, the cells were maintained in Dulbecco's modified Eagle's medium (DMEM, Solarbio Science & Technology, Beijing, China) supplemented with 10% fetal bovine serum (FBS, Gibco BRL, Gaithersburg, MD, USA), 100 U/mL penicillin, and 100 *μ*g/mL streptomycin (Shanxi MiniBio Technology Co., Ltd, Shanxi, China) in a 5% CO_2_ incubator at 37°C. The medium was replaced the next day.

### 2.5. Cytotoxicity of the Extracts with CCK-8 Assay

The relative survival rate of cells was detected and calculated by cell counting kit 8 (CCK-8) assay to indicate the cytotoxicity. RAW264.7 cells were seeded into 96-well plates at a density of 1 × 10^6^ cells/mL and cultured in a 10% FBS DMEM for 24 h. Following another 24 h treatment with the extracts at 0, 25, 50, 100, 200, and 400 *μ*g/mL, the supernatants were removed, and each well was washed with PBS before the addition of 10% FBS DMEM and 10 *μ*L CCK-8 reagent (Shanxi MiniBio Technology Co., Ltd, Shanxi, China). Cell viability was determined by measuring the absorbance at 450 nm using a microporous plate reader (Model 550; Bio-Rad Laboratories, Inc., Hercules, CA, USA) after an incubation period of 2 h at 37°C. The average optical density was determined by examining six wells per group.

### 2.6. The Effects of the Extracts on CD206, Arg-1, IL-1*β,* and iNOS Protein Expressions on M0/M1 Macrophages

The normal medium-treated cells were the M0 macrophages (resting macrophages) and the LPS-treated cells were the M1 macrophages (classic activated macrophages). The iNOS, IL-1*β*, CD206, and Arg-1 protein expressions were tested by Western blotting after the chaga extracts (chaga crude polysaccharides) were used at 25, 50, 100, and 200 *μ*g/mL (CCP25, CCP50, CCP100, and CCP200) on M0 and M1 macrophages separately. The treated cells (1 × 10^6^ cells/ml) were removed from the culture media and lysed with RIPA lysis buffer from Solarbio Science & Technology (Beijing, China) for 30 min. The protein concentrations were determined using a BCA Protein Assay Kit from Solarbio Science & Technology (Beijing, China). Samples containing 50 *μ*g of protein were resolved by 10% SDS-PAGE electrophoresis and transferred to polyvinylidene fluoride membranes (Millipore, Shanghai, China) in a buffer tank with platinum wire electrodes. After immersing the membranes in 5% nonfat dried milk (diluted in 0.1% (v/v) Tween-20 PBS) for 2 h at room temperature to block the nonspecific binding, the membranes were incubated overnight with a primary antibody against iNOS (Catalog No. 18985-1-AP, Proteintech, Wuhan, China) at 1 : 2000 dilution, a primary antibody against IL-1*β* (Catalog No. bs-0812R, Bioss, Beijing, China) at 1 : 1000 dilution, a primary antibody against CD206 (Catalog No. bs-21473R, Bioss, Beijing, China) at 1 : 1000 dilution, and a primary antibody against Arg-1 (Catalog No. 16001-1-AP, Proteintech, Wuhan, China) at 1 : 5000 dilution at 4°C. The membranes were washed four times (15 min each) and then incubated with the corresponding secondary IgG conjugated to HRP antibody (Catalog No. SA00001-2, Proteintech, Wuhan, China) at room temperature for 1 h. The results were finally analyzed by the Quantity One analysis system (Bio-Rad, Hercules, CA, USA). GAPDH at a dilution of 1 : 5000 (Catalog No. 10494-1-AP, Proteintech, Wuhan, China) was used as the internal loading control.

### 2.7. The Effects of the Extracts on IL-1*β*, TNF-*α,* and NO Levels on M0/M1 Macrophages

M0 macrophages (1 × 10^6^ cells/mL) and M1 macrophages (1 × 10^6^ cells/mL) were treated with CCP25, CCP50, CCP100, and CCP200 for 24 h separately. Cell supernatants were then harvested and centrifuged at 1,500 g for 10 min at 4°C. The IL-1*β* level was determined using an ELISA kit (Catalog No. MM-0040M1, Jiangsu Meimian Industrial Co., Ltd). The TNF-*α* level was determined using an ELISA kit (Catalog No. MM-0132M1, Jiangsu Meimian Industrial Co., Ltd). The absorbance was measured using a microplate reader (Model 550, Bio-Rad Laboratories, Inc.). Each sample underwent repeated testing three times.

The NO level was tested with the Griess assay. Nitrite, a stable end-product of NO metabolism, was measured using the Griess reaction. Culture media of the RAW 264.7 cells (100 *μ*L) was mixed with an equal volume of Griess reagent (Yantai Science & Biotechnology Co. LTD, Yantai, China), followed by spectrophotometric measurement at 540 nm (Model 550, Bio-Rad Laboratories, Inc.). Nitrite concentrations in the culture media were determined by comparison with a sodium nitrite standard curve. All experiments were repeated three times.

### 2.8. Statistical Analysis

The SPSS 19.0 software (IBM, Armonk, NY, US) was used for statistical analysis. All the data were expressed as mean ± standard deviation (SD) of the mean. A two-sided Student's *t*-test was used to analyze the differences between the two groups. One-way analysis of variance with Bonferroni's posttest was used when more than two groups were present. A *P* value of <0.05 was considered statistically significant.

## 3. Results

### 3.1. The Polysaccharides and Polyphenol Content

A total of 112.5 g of extracts was obtained from 1 kg of chaga, with an extraction rate of 11.3%. Using the phenol-sulfuric acid method, the content of polysaccharides in the extract was measured to be 13.7%, i.e., 100 g of the extract contained 13.7 g of polysaccharides. With Folin–Ciocalteu method, the results showed that 100 g extracts contained 1.9 g polyphenol.

### 3.2. The Cytotoxicity Results

CCK-8 results showed that the extracts at 400 *μ*g/mL inhibited the growth of RAW 264.7 cells (cell viability: (67.7 ± 4.7)%), which had a significant difference compared to the extracts at 0 *μ*g/mL ((100.0 ± 3.9)%, *P* < 0.001) and was unsuitable for further tests. The cell viabilities of the CCP25, CCP50, CCP100, and CCP200 were (103.0 ± 4.6)%, (98.2 ± 5.8)%, (98.6 ± 6.2)%, and (97.3 ± 4.7)%, respectively, which had no significant difference compared to the extracts at 0 *μ*g/mL and could be used for the following research.

### 3.3. The Results of the Extracts on CD206, Arg-1, IL-1*β*, and iNOS Protein Expressions in M0 Macrophages

Figures 4(a)–4(c) show the CD206, Arg-1, IL-1*β* and iNOS protein expression of CCP25, CCP50, CCP100, CCP200 on M0 macrophages. The analyses in Figures 4(d) and 4(e) indicated that compared to M0, CCP25 and CCP50 decreased CD206 expression significantly (*P* < 0.001 and *P*=0.007), and CCP50 decreased Arg-1 expression significantly (*P* < 0.001). In Figures 4(f) and 4(g), we could see that compared to M0, CCP50 and CCP100 significantly increased IL-1*β* expression (*P*=0.003 and *P*=0.005), and CCP 25 and CCP 200 increased iNOS expression significantly (both: *P* < 0.001).

Further analyses showed that the increased effect on IL-1*β* expression of CCP100 was better than CCP50 significantly (*P*=0.033), and the increased effect on iNOS expression of CCP200 was better than CCP25 significantly (*P*=0.008).

### 3.4. The Results of the Extracts on CD206, Arg-1, IL-1*β,* and iNOS Protein Expressions in M1 Macrophages

Figures 5(a)‒5(d) show that the protein expression results of CD206, Arg-1, IL-1*β,* and iNOS after M1 macrophages were intervened with CCP. Compared with the M0 macrophages, CD206 and Arg-1 protein expression decreased (*P* < 0.001, *P*=0.001) in Figures 5(e) and 5(f), while IL-1*β* and iNOS protein expression of M1 macrophages significantly increased (*P*=0.005, *P* < 0.001) in Figures 5(g) and 5(h).

Compared with the M1 macrophages, significantly increasing effects of CCP50, CCP100, and CCP200 on CD206 expression could be seen in Figure 5(e) (*P*=0.002, *P* < 0.001 and *P* < 0.001). Among the above three concentrations, CCP200 showed its best effects compared with CCP50 (*P*=0.003) and CCP100 (*P*=0.008).

Also compared with the M1 macrophages, CCP25, CCP100, and CCP200 increased Arg-1 expression significantly (*P*=0.001, *P*=0.019 and *P* < 0.001), and CCP200 was better than CCP25 (*P* < 0.001) and even better than M0 macrophages (*P* < 0.001).

Compared with the M1 macrophages again, CCP200 decreased IL-1*β* and iNOS expression significantly (*P*=0.037 and *P* < 0.001*P* < 0.001) and CCP100 decreased iNOS significantly (*P*=0.004). The decreasing effect on iNOS of CCP200 was better than CCP100 (*P*=0.010).

### 3.5. The Results of the Extracts on IL-1*β*, TNF-*α,* and NO Levels in M0 Macrophages

Compared with the NO level of the M0 macrophages ((2.7 ± 0.6) *μ*M), CCP50 ((9.3 ± 3.2) *μ*M), CCP100 ((14.2 ± 3.5) *μ*M), and CCP200 ((18.6 ± 2.1) *μ*M) all showed significant increasing effects on NO production (*P*=0.025, *P*=0.005 and *P* < 0.001). The increased NO production of CCP200 was significantly higher than CCP50 (*P*=0.014).

Compared with the TNF-*α* level of M0 macrophages ((452.9 ± 36.3) pg/mL), both CCP100 ((570.5 ± 21.0) pg/mL) and CCP200 ((606.5 ± 86.1) pg/ml) showed significant increasing effects on TNF-*α* level (*P*=0.008 and *P*=0.047).

### 3.6. The Results of the Extracts on IL-1*β*, TNF-*α,* and NO Levels in M1 Macrophages

Compared with the M0 macrophages, the NO production of M1 macrophages increased from (2.7 ± 0.6) *μ*M to (86.9 ± 0.9) *μ*M (*P* < 0.001), promoted IL-1*β* level in macrophages from (90.7 ± 6.7) pg/mL to (146.2 ± 7.9) pg/mL (*P* < 0.001), and elevated TNF-*α* content from (452.9 ± 36.3) pg/mL to (522.2 ± 45.7) pg/mL. Results are shown in Figures 6(a)–6(c).

In Figure 6(a), CCP25, CCP50, CCP100, and CCP200 all had significant effects on decreasing NO production in M1 macrophages (All: *P* < 0.001). The decreasing effects of CCP200 showed significantly better results compared with CCP25 (*P*=0.015) and CCP50 (*P*=0.026).

Compared with the IL-1*β* level of M1 macrophages in Figure 6(b), CCP at four tested concentrations all showed the decreasing effects, but only CCP100 ((109.5 ± 9.2) pg/mL) and CCP200 ((114.0 ± 10.0) pg/mL) showed significant effects (*P*=0.006 and *P*=0.012).

Finally, on TNF-*α* level in Figure 6(c), CCP200 showed its decreasing effects significantly ((350.8 ± 6.9) pg/mL, *P*=0.003) when compared with M1 macrophages.

## 4. Discussion

Polysaccharides are among the most important members of the biopolymer family. They are natural macromolecules composed of monosaccharides. To date, more than 300 kinds of natural polysaccharide compounds have been identified. They are present in plants, microorganisms, and engage in a variety of physiological functions [31]. The crude extracts of the medicinal mushroom chaga have been used as effective traditional medicine to treat malicious tumors, gastritis, gastric ulcers, and other inflammatory conditions [32]. Our literature research in Figure 1 supported that among the extracts from chaga, polysaccharides are major bioactive components that possess antitumor, hypoglycemic, and anti-inflammation activities [33]. As we mentioned before, cancer and diabetes are both regarded as immunology-related diseases [6, 7]. Antitumor and hypoglycemic mechanisms related to immunomodulatory activities of chaga polysaccharides are further summarized in Figure 2.

Figure 2 shows that antitumor activities of chaga polysaccharides are achieved through multiple signals including but not limited to the activation of the nod-like receptor family protein 3 (NLRP3) inflammasome, nuclear factor *κ*appa B(NF-*κ*B)/mitogen-activated protein kinases (MAPK) pathway, liver kinase B 1(LKB1)/AMPK pathway, and the promoted effects on NO, TNF-*α,* and IL-1*β* level via above signals and immuno-stimulating effects [15–21]. Figure 2 also shows that *in vivo* hypoglycemic activities of chaga polysaccharides are confirmed by depressing oxidative stress, NF-*κ*B/transforming growth factor (TGF)-*β* pathway, and PI3K/Akt pathway. Accordingly, their hypoglycemic activities are correlated with the inhibition of TNF-*α*, IL-1*β*, NF-*κ*B, and ROS level [9–11]. Based on the above discussion, it seemed that chaga polysaccharides have bilateral immunomodulatory effects on TNF-*α*, IL-1*β*, etc. in the face of cancer and diabetes.

Water extraction and ethanol precipitation are popular methods to obtain crude polysaccharides from many fruiting bodies of mushrooms, such as *Coriolus versicolor* [34] and *Grifola frondosa* [35]. It was reported that *I. obliquus* polysaccharides could be initially purified via precipitation from an aqueous extract with 80% alcohol [36]. The chaga crude polysaccharides were obtained in our research with the above similar method and were further studied on macrophages at M0 resting condition and LPS-activated M1 subtype.

As pivotal immune stromal cells in the tumor microenvironment (TME), macrophages are extensively heterogeneous and exert both antitumor and protumor functions [37]. Tumor-associated macrophages (TAMs) are the critical components of tumors and play an important role in the development of the immunosuppressive TME. It was reported that the transition of TAMs from M2 to M1 is crucial for the immunotherapy of gastric cancer [38]. Some related research showed that polysaccharides isolated from the fruiting body of chaga was capable of promoting NO/ROS production, TNF-*α* secretion, and phagocytic uptake in macrophages RAW264.7 cells [16]. Figure 2 also shows that anticancer activities of chaga polysaccharides were related to increased NO, ROS, and TNF-*α* levels on macrophages [15, 16]. Our research confirmed for the first time *in vitro* that the elevated NO, TNF-*α,* and IL-1*β* levels of chaga crude polysaccharides might related to their activities in increasing M0 to M1 polarization and decreasing M2 polarization.

It was reported that the chaga polysaccharide can ameliorate azoxymethane/dextran sulfate sodium-induced colitis-associated cancer in mice [17]. Colon cancer is a common and deadly human digestive tract malignant tumor with a poor prognosis [39]. Triptolide is extracted from the traditional Chinese medicine *Tripterygium wilfordii*. Related research showed that triptolide-educated colon cancers retarded the macrophages' polarization to anti-inflammatory M2 status by decreasing the expression of Arg-1 and CD206, the markers of M2 polarization [39]. Could chaga polysaccharide exert its anticancer activity by promoting M0 to M1 subtype and decreasing M0 to M2 polarization? Further *in vivo* research should be conducted.

T2DM is characterized by low-grade chronic inflammation and metabolic dysfunction, which is observed in all tissues involved in energy homeostasis. A substantial body of evidence has established an important role for macrophages in these tissues during the development of T2DM [40]. Some related *in vivo* research demonstrated that hyperglycemia could polarize macrophages toward M1 via overproducing ROS under inflammatory condition [41]. An animal study showed that the mechanism of fasudil on the diabetic nephropathy progression might be associated with its induction of M2 polarization and the reduction of M1 polarization and inflammation [42]. A novel macrophage-regulating drug was reported to accelerate wound healing in a diabetic mouse model by decreasing M1 activity and enriching M2 populations. Furthermore, the efficiency of this macrophage-regulating medicine was confirmed in a multicenter, evaluator-blinded, phase 3 randomized clinical trial, which was performed across the US, China, and Taiwan [43].

In recent years, research on M1/M2 differentiation of chaga extract has been explored, such as inonotsuoxide B, a tetracyclic triterpenoid extracted from chaga, was reported to have a regulation effect on macrophage polarization [44]. To the best of our knowledge, our current work was the first study on the effect of chaga crude polysaccharides on regulating M1 to M2 phenotype. Our previous research showed that the protective effects of two safflower-derived compounds on hyperglycaemic stress-induced renal podocyte apoptosis via modulating macrophage M1 to M2 polarization [23]. We will try a study on M1/M2 subtype on diabetic animal model with chaga-purified polysaccharide in our following research.

In Table 1, it was interesting to see that when tested on resting the macrophage, CCP50 targeted both the markers of M1 and M2 including CD206, Arg-1, and IL-1*β* to produce NO. CCP200 increased iNOS expression to elevate NO and TNF-*α* level. When tested on M1, CCP100 and CCP200 had effects on the markers of M1 and also M2, but CCP25 and CCP50 only increased the protein expressions of M2. The potential reason of the above results might be that the other active ingredients such as polyphenols and flavonoids also extracted simultaneously when aqueous extraction and alcoholic precipitation was used mainly for polysaccharides extraction [45]. Our research already confirmed that in addition to polysaccharides in the extracts, polyphenols were also present [46].

Some findings indicated that chaga polysaccharides exert immune-enhancing activity and other components in chaga also displayed antitumor activity [47]. Do different components have different effects on macrophage polarization? Further studies should probably focus on some purified compounds and their relationships with macrophage differentiation, such as inonotsuoxide B. The antitumor activity of inonotsuoxide B [48] and its regulation on macrophage polarization through sirtuin-1/endoplasmic reticulum stress axis [44] was explored.

In recent years, the structure determinations of chaga polysaccharides and their antitumor and antidiabetic research have already made some progress. The structure characterization and hypoglycaemic activities of two polysaccharides from *I. obliquus* were reported recently [49]. A novel water-soluble polysaccharide was isolated and purified from chaga. Its chemical characteristics and antitumor, immunoregulatory activity were also investigated [50]. With the help of experts in the chemical structure analysis, the structural characterization and immune activity screening of polysaccharides with different molecular weights [51] from chaga crude polysaccharides is being studied by our research team. The relationships of purified polysaccharides and their immunomodulatory roles related to macrophage polarization could have prospects.

## 5. Conclusions

Chaga, a parasitic fungus, has drawn more interest in recent years for its multiple pharmacological actions. According to our literature research, chaga polysaccharides play important roles in antitumor and antidiabetic activities. The resting macrophages can be polarized to M1 or M2 subtype, which play different immunomodulatory roles when macrophages exert anticancer and antidiabetic activities. Our current *in vitro* research suggested that the bilateral effects of the chaga extracts on TNF-*α*, IL-1*β,* and NO level on M0/M1 macrophages might be related to its contained polysaccharides and chaga polyphenols. Further anticancer and antidiabetic research of purified chaga polysaccharide and polyphenol related to macrophage polarization should be conducted *in vivo*.

## Figures and Tables

**Figure 1:** The articles of chaga and its active ingredients in the research of different diseases. (a) The articles of chaga. (b) The articles of chaga polysaccharides. (c) The articles of chaga polyphenols. Note: the literature survey was conducted over the last 10 years (2012–2021). Wanfang, Wanfang database; CNKI, China National Knowledge Infrastructure.

**Figure 2:** Antidiabetes and anticancer research of chaga polysaccharides based on immune-related signaling pathways. Abbreviations: AMPK, adenosine monophosphate-activated protein kinase; Akt, protein kinase B; AOM, azoxymethane; Bax, Bcl-2-associated X protein; Bcl-2, B-cell lymphoma 2; C/EBP*α*, CCAAT/enhancer-binding protein *α*; COX-2, cyclooxygenase-2; DKD, diabetic kidney disease; DM, diabetes mellitus; DSS, dextran sulfate sodium; ERK, extracellular signal-regulated kinase; GLUT4, glucose transporter protein 4; HFD, high fat diet; IL-1*β*, interleukin-1*β*; IL-2, interleukin-2; IL-18, interleukin-18; JNK, c-Jun N-terminal kinase; LKB1, liver kinase B 1; MAPK, mitogen-activated protein kinases; MMP-2, matrix metalloprotein-2; MMP-7, matrix metalloprotein-7; MMP-9, matrix metalloprotein-9; mTOR, mammalian target of rapamycin; NF-*κ*B, nuclear factor *κ*appa B; NLRP3, the nod-like receptor family protein 3; NO, nitric oxide; PARP, poly ADP-ribose polymerase; PI3K, phosphatidylinositol 3 kinase; PPAR*γ*, peroxisome proliferator-activated receptors *γ*; T2DM, type 2 diabetes mellitus; TGF-*β*, transforming growth factor-*β*; TNF-*α*, tumor necrosis factor-*α*; STZ, streptozotocin.

**Figure 3:** Extraction flowchart.

**Figure 4:** Effects of CCP on CD206, Arg-1, IL-1*β,* and iNOS protein expressions in M0 macrophages. (a) CD206 protein expressions. (b) Arg-1 and IL-1*β* protein expressions. (c) iNOS protein expression. The results of CD206, Arg-1, IL-1*β,* and iNOS protein expressions were represented in (d), (e), (f), and (g), respectively. All results were expressed as a ratio with respect to M0 and represented as the mean ± SD in triplicate. ^#^*P* < 0.05, CCP versus M0. CCP, chaga crude polysaccharides; CCP 25, CCP at 25 *μ*g/mL; CCP 50, CCP at 50 *μ*g/mL; CCP 100, CCP at 100 *μ*g/mL; CCP 200, CCP at 200 *μ*g/mL; CD206, mannose receptor; Arg-1, arginase-1; IL-1*β*, interleukin-1*β*; iNOS, inducible nitric oxide synthase; M0, resting macrophages.

**Figure 5:** Effects of CCP on CD206, Arg-1, IL-1*β,* and iNOS protein expressions in M1 macrophages. (a) CD206 protein expressions. (b) Arg-1 protein expressions. (c) IL-1*β* protein expressions. (d) iNOS protein expression. The results of CD206, Arg-1, IL-1*β,* and iNOS were represented in (e), (f), (g), and (h), respectively. All results were expressed as a ration with respect to M0 control and represented as the mean ± SD in triplicate. ^#^*P* < 0.05, M1 versus M0. ^*∗*^*P* < 0.05, CCP versus M1. CCP, chaga crude polysaccharides; LPS, lipopolysaccharide; CCP 25, CCP at 25 *μ*g/mL; CCP 50, CCP at 50 *μ*g/mL; CCP 100, CCP at 100 *μ*g/mL; CCP 200, CCP at 200 *μ*g/mL; CD206, mannose receptor; Arg-1, arginase-1; IL-1*β*, interleukin-1*β*; iNOS, inducible nitric oxide synthase; M0, resting macrophages; M1, classic activated macrophages.

**Figure 6:** Effects of CCP on nitric oxide production, IL-1*β*, and TNF-*α* level in M0 and M1 macrophages. (a) Nitrite (nitric oxide production) levels. (b) IL-1*β* levels. (c) TNF-*α* levels. Values were expressed as the mean ± SD of the mean (*n* = 3). ^#^P < 0.05, M1 versus M0. ^*∗*^*P* < 0.05, CCP versus M1. CCP, chaga crude polysaccharides; LPS, lipopolysaccharide; CCP 25, CCP at 25 *μ*g/mL; CCP 50, CCP at 50 *μ*g/mL; CCP 100, CCP at 100 *μ*g/mL; CCP 200, CCP at 200 *μ*g/mL; IL-1*β*, interleukin-1*β*; TNF-*α*, tumor necrosis factor-*α*; M0, resting macrophages; M1, classic activated macrophages.

**Table 1:** Comparison of CCP at different concentrations on M0 to M1/M2 and M1 to M2 regulation.

Regulation on macrophage polarization	The markers of M1 and M2	CCP25	CCP50	CCP100	CCP200
M0 to M1/M2 (CCP on M0 macrophages	CD206	^#^	^#^		
	Arg-1		^#^		
	IL-1*β*		^#^	^#^	
	iNOS	^#^			^#^
M1 to M2 (CCP on M1 macrophages)	CD206		^*∗*^	^*∗*^	^*∗*^
	Arg-1	^*∗*^		^*∗*^	^*∗*^
	IL-1*β*				^*∗*^
	iNOS			^*∗*^	^*∗*^

Notes: ^#^ represented as a significant difference compared to M0 macrophages. ^*∗*^Represented as a significant difference compared to M1 macrophages. M0, resting macrophage; M1, classic activated macrophage; M2, alternative activated macrophage; CCP, chaga crude polysaccharides; LPS, lipopolysaccharide; CCP25, CCP at 25 *μ*g/mL; CCP50, CCP at 50 *μ*g/mL; CCP100, CCP at 100 *μ*g/mL; CCP200, CCP at 200 *μ*g/mL; CD206, mannose receptor; Arg-1, arginase-1; IL-1*β*, interleukin-1*β*; iNOS, inducible nitric oxide synthase.

## Data Availability

The readers can access the data supporting the conclusions of the study from Figures 1–6 and Table 1. All those figures and tables are included within the manuscript. All authors declare that the data of the manuscripts can be verified from the results of the article, be replicated in the analysis, and be conducted in secondary analyses.
